This article has been retracted.

# Visual Communication Design Model for New Media and Public Health Environment and New Communication Mode

**DOI:** 10.1155/2022/1177677

**Published:** 2022-09-25

**Authors:** Ke Wang, Caiyuan Kuang

**Affiliations:** Jinling Institute of Technology, Nanjing 211169, China

## Abstract

When we examine the development history of visual transmission design, we can see that media technology application and visual transmission design innovation are frequently intertwined. The relevant work outcomes attained during the process of art design practice typically exhibit the traits of dynamic and dynamic performance with a clear degree of expression, against the backdrop of the practical advancement and widespread use of developing media technology. In light of the influence of new media art, it is essential to understand the development trend of art design in order to perform well in visual transmission design. The audience will be given access to more varied and richer visual transmission information thanks to the wise deployment of multimedia techniques. This work develops a three-dimensional picture reconstruction algorithm based on the visual transmission phenomenon. The relative error, matching degree, and signal-to-noise ratio were chosen as evaluation indices. Three sets of tests were conducted to determine how noiseless image, noisy image, and various sampling frequencies affected the quality of the reconstructed image. The testing results demonstrate that the three-dimensional picture rebuilding system has a 22.34% higher antinoise ability and has a significantly superior overall effect than the conventional three-dimensional image rebuilding system. It offers greater practical application value and does a decent job of keeping image details and edges.

## 1. Introduction

In this era of information explosion and resource sharing, we started to consider how to acquire more information more quickly and effectively in the simplest way, as well as how to fully and sustainably utilize our shared resources [1]. The development of science and technology in the modern era has given rise to new media, which also expands the communication channels available for artistic expression. The great speed and directness brought by developing media, however, are not well understood by most people because they have not been around for a very long period [2]. As human spiritual civilization advances and gradually enters the period of new media, substantial worry has been raised about the significant influence that this development will have on contemporary art and design. The traits of contemporary art and design practice work in the age of developing media are also continually emphasized [3]. According to the evolving media theory, there will inevitably be a movement toward a diversity of visual transmission design form and design content. Therefore, if we want to ensure that the visual design conforms to the current trend of the times, we must actively innovate the elements of visual transmission and enrich the information conveyed by the design. With the progress of emerging media art design, designers also need to optimize the work of integration, connection, and interaction in visual transmission design [4]. When we contrast the visual transmission design under the influence of emerging media art design with the traditional art design, we can see that the form of emerging media art design has the ability to convert the traditional static art design effect into the dynamic art design effect and to incorporate the concept of time into the design in the art works [5].

The dynamic expression of graphic pictures and text is one of the dynamic visual design aspects of visual transmission from the standpoint of design elements. The movement of the design elements should be taken into account during the design phase in addition to their visual appearance [6]. The designer's thinking must change for the process to effectively transmit information, and the design and creation are viewed from a multidimensional and three-dimensional perspective. The “new communication” and “new language” of the visual design already present in emerging media, as well as an in-depth examination of new modes of expression and particular applications in emerging media, should be the focus of visual transmission design under emerging media technology rather than simply remaining in the traditional design under the influence of technology [7]. In this paper, a compressed sensing 3D image rebuilding algorithm based on visual transmission effect is formed, and experiments are carried out from three evaluation indicators, which theoretically improves the practical application value.

Traditional visual transmission usually reflects the visual impact to attract people's attention through color matching, image splicing, text design, and composition diversification to achieve the purpose of conveying information. The means used by emerging media works will be relatively novel and diverse. It reflects the vividness of visual transmission through dynamic images and video broadcasting. It uses the processing of dynamic images to achieve various special effects in line with the scene to stimulate people's eyeballs and opens people's ears with a variety of music and dubbing forms. More works allow people to explore the mysterious parts of the works through the touch terminal. Visual transmission itself has been constantly updated and developed. Both the plane and the display have injected scientific and technological power and updated the media [8]. These new forces have not only enriched the forms of expression of visual transmission but also enriched the content of expression. They have also narrowed the cognitive distance between people and information and made people pay more attention to and favor emerging media art in their lives. The main contributions of this paper are as follows:

1. Based on the image enhancement theory, starting from the visual characteristics of the human eye, the discrete entropy, contrast sensitivity, resolution, and other indicators of the image are improved, and the visual transmission effect of the image is optimized
2. Apply image classification technology to retrieve cases similar to sample images and find similar areas to distinguish plagiarized designs, so as to protect the designer's patents and homogenized design issues

## 2. Related Work

Under the influence of emerging media technology, the creative space of art design has also undergone great changes, and the visual thinking of art designers has also undergone great changes. Moreover, the progress of emerging media art design has also brought greater challenges to aesthetic concepts and artistic values. Osborn analyzed the in-depth development history of the fast evolving multimedia technology in the modern period and talked about the benefits it brings to business. It also explains the meaning of visual culture and the impact of new technologies on people's ways of thinking and living [9]. Focusing on the fundamental techniques and concepts of visual design, Piegl et al. demonstrate how designers can use these design abilities to produce original choices that result in effective visual information exchange [10]. There have also been more subdivided studies between emerging media and visual transmission in China. In his edited “Visual Communication and Media Application,” Zheng et al. expounded the changing relationship between media and visual transmission, as well as the platform and ideas that media application provides for visual transmission [11]. Li speculates on the new trend of media progress in the digital age and proposes the new term “transmedia” and its existing form and characteristics and focuses on the inspiration of digital media in creative thinking [12]. According to Myers, the formation of new design languages has been facilitated by the rapid development of digital multimedia technology, which has improved visual transmission design manifestations from static presentation to dynamic presentation [13]. Lee and Kim pointed out that with the support of the Internet and computers, graphic works designed through visual transmission show more and more rich characteristics, especially now that many graphic design software can directly help authors design complex and changeable patterns [14]. Carroll a believes that in the process of digital media design, the unique characteristics of sound, light, electricity, and human-machine interaction of digital media are used to more effectively achieve the purpose of disseminating information. It can be considered that the connotation and characteristics of emerging media art design are the further enrichment of visual transmission art design [15]. Cracken proposed specific strategies to improve the visual transmission design effect under the emerging media background and carried out a brief analysis and discussion from two aspects, aiming to provide empirical reference for researchers in related fields [16]. In terms of visual transmission image processing technology, Peng and Li took the initial image as the basic image and the detail image through guided filtering, equalized the basic image with the histogram with contrast limitation, fused the processed two images, and obtained the final image with enhancement processing [17]. Fan said that as a part of modern design, visual transmission design is destined to serve production and consumption. If you want to stand out from many similar competitors, it is far from enough to faithfully describe the content of information. Therefore, a creative visual image must become a visual transmission [18].

## 3. Visual Communication 3D Image Design

The application and popularization of modern technology and the introduction of modern scientific and technological means also promote the continuous updating and expansion of artistic design concepts and disciplines. As a new subject, media art design is also born from this application and also shows great progress potential and market space. Media art design uses various media centered on computers as tools to design works. It covers a series of cultural and creative forms that comprehensively apply various modern media, high-tech means, and modern design language, such as digital animation, digital images, photoelectric integrated media, and interactive art design. Visual transmission technology [19], which has technical applications in a variety of industries, processes images using multimedia technology. With the emergence of developing media, the traditional visual transmission design has changed from the straightforward transmission of visual information to a multisensory experience that includes touch and hearing. This multisensory blending and communication that goes beyond eyesight gives the audience a more holistic and humanized experience [20]. The system is composed of three components, namely, an image analysis module, an image preprocessing module, and a 3D visualization module, as shown in Figure 1.

Although the concept and some of the content are determined during the visual design process, it is like providing a framework. The most crucial factor, however, is how the designer employs various components to complete this framework, enhance the design content, and include more pertinently into the design scheme. Visual transmission design often focuses on informing the audience of information, and in this process, media technology is crucial to accomplishing a goal of communicating. The media and visual transmission art design can have some interactive relationships, though, in that the media can employ visual transmission art design to influence and effectively encourage the growth of developing media. The recipient's feelings should be taken into account for picture design processing at any point, as indicated in Figure 2, while designing a new media in addition to adhering to the traditional aesthetic concept.

A vivid graphic can directly transmit the information to be transmitted and has the characteristics of easy identification and memory. Therefore, visual transmission design can be completely freed from the shackles of language and words and can be used all over the world. Due to the continuous progress of various emerging media technologies, we need to transform visual transmission design from the traditional level. Visually, it is divided into from static to dynamic and from two-dimensional to three-dimensional. Here, the technical structure of 3D visualization is introduced to verify the application of a large number of new technologies in the process of visual transmission design (Figure 3). Among them, let the audience experience more levels of emerging media technology, so as to obtain more accurate, efficient, and diversified information. At the same time, this new form of visual transmission design can make the information leave a deeper impression in the audience's mind, so that the information can be communicated better.

## 4. Algorithms and Experiments

### 4.1. Introduction to 3D Reconstruction Algorithms

Aiming at the shortcomings of the traditional image compression sensing rebuilding algorithm's poor visual transmission effect and low imaging quality, the image segmentation theory is introduced into the compressed sensing image rebuilding. Combined with the advantages of curvelet transform, which is suitable for expressing edge detail information and curve information, the image is sparsely represented by curvelet transform, and an image compressive sensing image rebuilding algorithm based on visual transmission effect is formed. In digital image processing theory, the discrete wavelet transform (DWT) algorithm is introduced, and the formula is as follows.

(1) $$\begin{array}{c} \delta =\sqrt{\text{In}\left|\frac{L_{k}}{i}\right|}, \end{array}$$

where *L*_*k*_ represents the wavelet packet decomposition coefficient.

For wavelet transform, it is necessary to define a scale function and denote the scale function as *φ*(*t*) and its Fourier transform as *ϕ*(*w*). The Fourier transform of *φ*(*t*) in formula (1) is *ϕ*(*w*), and then the expression of the real part of the filter bank is

(2) $$\begin{array}{c} \varphi \left(t\right)=\sqrt{2}\underset{n}{\sum }h_{0}\left(n\right)\varphi \left(2t-n\right), \end{array}$$

(3) $$\begin{array}{c} \phi \left(t\right)=\sqrt{2}\underset{n}{\sum }h_{0}\left(n\right)\phi \left(2t-n\right). \end{array}$$

On the basis of wavelet transform, the main purpose of detecting the visual transmission edge of an image is to effectively identify the edge details in the image and compare the detected edge information with the corresponding neighborhood information. If the neighborhood information does not belong to the edge component, the detection is stopped, and a binarized edge image is established. Use “0” for nonedge component and “1” for edge component. Image edge detection can not only effectively identify the edge information in the visual transmission image but also accurately divide different subblocks. The image threshold is calculated by the following formula:

(4) $$\begin{array}{c} \beta =\varepsilon \sqrt{2I\text{n}F}. \end{array}$$

Assuming that the contour point in the image of the object has a set of contour lines connected to it, the layered write operation is carried out on the image data field, and the definition is based on the contour point as the starting point. The 3 × 3 field of the current pixel is then searched counterclockwise. Take the first nonzero point encountered during the search as the next contour point. Then, continue searching with it as the starting point until there are no nonzero points in the field. The state function *T*(*a*, *b*, *c*) of each voxel (*a*, *b*, *c*) in the data is

(5) $$\begin{array}{c} T\left(a,b,c\right)=\left\{{}_{0,\left(a,b,c\right)\in \text{line}.}^{-1,\left(a,b,c\right)\notin \text{line},}\right. \end{array}$$

In the process of actual operation, the characteristics of the image containing complex information and the ambiguity contained in the image in the process of image processing are comprehensively considered, which promotes the visual effect of the entire image to be significantly improved. The fitness values of different particles are calculated separately, the candidate positions are clarified, and the tabu table is updated at the same time. Since the recognition efficiency and different data volumes are not compared and analyzed in the previous formula, the application effect of the design method in all scenarios cannot be guaranteed. In the future, supplementary analysis will be carried out to better improve the visual transmission effect.

In the same way, combining the wavelet decomposition method with the improved global threshold algorithm, the original noise image is wavelet decomposed, the noise level of different subbands, and the edge strength of the image is calculated, so as to obtain the adaptive threshold. The expression of the filter bank of its conjugate part can be obtained:

(6) $$\begin{array}{c} \varphi_{g}\left(t\right)=\sqrt{2}\underset{n}{\sum }g_{0}\left(n\right)\varphi_{g}\left(2t-n\right), \end{array}$$

(7) $$\begin{array}{c} \phi_{g}\left(t\right)=\sqrt{2}\underset{n}{\sum }g_{1}\left(n\right)\phi_{g}\left(2t-n\right). \end{array}$$

In time-based design, each action or scene consists of a continuous, time-controlled sequence that forms a timeline, or narrative structure, and the dynamic text on the screen is based on twenty-four frames per second. The speed display makes the still image dynamic through the change of the time series, and because of the movement of the text, the temporary reading is caused, and an information impression is formed in people's minds through vision. Therefore, designers should consider how to effectively transmit information through the movement of fonts in a short period of time when creating. The formula is as follows:

(8) $$\begin{array}{c} f\left(\alpha \right)=\alpha_{k}\cdot H_{k}T+k_{0}. \end{array}$$

In the formula, *f*(*α*) represents the data discriminant model of the hyperplane, *α*_*k*_ represents the parameter features of the hyperplane, *H*_*k*_*T* represents the class label of the distance matrix, and *k*_0_ represents the degree of separation of the samples.

After completing the 3 × 3 domain search, it is found that the contour that is visually continuous but discontinuous in the contour map cannot be accurately obtained, especially the closed contour with obvious features. Therefore, the algorithm is extended to continue searching in the 4 × 4 field. If the initial starting point is encountered in the search process, the previous point will be connected with it to form a closed contour. If new nonzero points are encountered, the search will continue, and the nonzero points obtained by the search will be connected to obtain as many closed contours as possible to improve the matching efficiency of the algorithm.

In order to have a clear quantitative standard for the effect of visual transmission, this paper uses discrete entropy *H*(*p*), contrast *Q*, and sharpness *C* as evaluation indexes, and their respective definitions are as follows:

(9) $$\begin{array}{c} H\left(p\right)=-\underset{i=0}{\sum }p\left(i\right)\log_{2}p\left(i\right), \end{array}$$

(10) $$\begin{array}{c} Q=\sqrt{{RF}^{2}+{CF}^{2}}, \end{array}$$

(11) $$\begin{array}{c} C=\underset{\sigma }{\sum }\sigma^{2}\left(i,j\right)P_{\sigma }\left(i,j\right). \end{array}$$

Each element can be saved as a characteristic in the mass center by assembling these movable optical components. The distance between each image's visual connection area and quality center is calculated using the proficient visual data, and the statistical results are presented graphically and saved in the classifier.

### 4.2. Experiment

In this article, the effectiveness of the graphics and image processing approach is examined through comparative tests in order to compare its practical applicability. In this case, the experimental data set's many pertinent parameters are simultaneously specified as an image data set is first created. The remaining images are utilized as the test library, and 200 images are then selected at random as the training library from the dataset. The registered images can preserve many aspects under various resolution features by extracting image contours. The Fourier feature matching algorithm is used to match the corresponding contours in different images, and the matching point pairs are obtained, which are used as the mapping points for the next image registration: image after alignment. In order to achieve multiview image registration, the transformation relationship between different images must be found. This method can clearly describe the contour features and detailed information of the image, as shown in Figure 4.

When thresholding the visual transmission image, part of the image information will be lost. At the same time, the image decomposition will also be affected, which will cause the loss of detail information of adjacent pixel blocks. Therefore, a pixel area of *n* × *n* is selected, and discrete wavelet transform is performed on different pixel blocks in the area. This is because the proposed method denoises the image before the image contrast enhancement, which lays a solid foundation for the subsequent contrast enhancement processing, which makes the enhancement effect and visual effect obtained by the proposed method significantly better (see Figure 5).

The likelihood of problems in the visual transmission design is typically higher when the content is relatively simple. This results in a situation where the content is similar in the visual transmission design, which will negatively affect the visual transmission design's ability to develop in the future. Designers must take into account the materials of the art design and the novelty of the content when designing in this context because the new media art design has a certain impact and influence on the traditional visual transmission design. This will enable the visual transmission design to work within the art design. This area is capable of receiving more fresh design concepts.

Since the image is obtained using 3D image mapping in the actual scene, some grayscale information will be lost throughout the acquisition process, leading to erroneous and blurry information. Image reconstruction heavily relies on sparse transformation and blur recognition. It has been frequently utilized in image processing to alter images sparsely using the curvelet approach. The transform basis is also fixed in the case of the conventional curvelet transform, which can only extract a small amount of directional information. As a result, it is impossible to entirely suppress the image's noise while maintaining its edge information. When evaluating the parameter attributes, it is crucial to examine how the method's critical parameters—such as the feature space's distribution law and the dictionary space's storage capacity—affect computer graphics and image processing performance (see Table 1).

Making sure the design scheme is beautiful, adding more pertinent aspects, and giving as much thought as you can to the content associated with the design theme are all crucial steps in the design process of new media art. In the field of image processing, a color space refers to a mathematical model that can provide a suitable color description for image processing. The visual transmission using the new media platform not only has a large amount of information and high timeliness, but more importantly, the visual transmission of the new media technology is flexible, has a wide radiation range, and is green. The information conveyed through the new media can be easily modified and improved at the first time, and the information will also be transformed synchronously from different terminals. The 3D image reconstruction system's rebuilding time and speedup are shown in Table 2 for various situations. The lengthening of the 3D picture reconstruction time of the two systems is caused by the enhancement of voxel division accuracy to varied degrees. Additionally, the speedup impact becomes more pronounced with an increase in voxel division precision as the speedup ratio increases.

A high-quality 3D image reconstruction system must guarantee high reconstruction accuracy while also guaranteeing high reconstruction effectiveness. The reconstruction accuracy and image quality of the experimental items that the two algorithms were able to reconstruct are shown in Table 2. When employing the system described in this research to reconstruct 3D images of objects, accuracy is greater than 95.6%, and rebuilding accuracy and clarity are much higher than when using RGB, according to an analysis of Table 2. Additionally, picture B's rebuilding accuracy is higher than image A's, showing that the system in this study can not only successfully reconstruct the three-dimensional image of the item but also that the rebuilding accuracy increases with image size to investigate the impact of various sample rates on the accuracy of image reconstruction. The shift independent discrete cosine (SID) approach and the patch-based directional (PBD) method's relative L2 error (rlne) of MRI images were as follows. The findings of the comparison are displayed in Figures 6–8.

In Figure 6, the relative error is represented by the ordinate, and the abscissa in the image represents the sample frequency, which is 0.32, 0.21, 0.12, 0.25, and 0.54, respectively. By way of illustration, consider Figure 6, where the relative inaccuracy of Sid and PBD is clearly higher than that of GPB. The local relative error can reach 0.010 when the sample frequency is 0.33. The theory of picture segmentation is incorporated into the compression sensing image reconstruction due to the drawbacks of the conventional curvilinear transform. An image compression sensing image rebuilding algorithm based on the curvilinear transform of image segmentation is proposed in order to suppress the image noise and preserve the edge information. This is in addition to the benefits of the curvilinear transform, which is suitable for expressing the edge detail information and curve information.

In the era of printing media as the main information communication method, visual transmission design is equivalent to graphic design. With the progress of technology and the diversification of contact forms, people have entered the era of digital information communication, and the field of visual transmission design has been broadened. In Network, multimedia, etc., digital media design becomes the new means of communication. Modern visual transmission design presents a multidimensional trend. Traditional graphic design is limited by print media, and the creative space is mainly concentrated in the plane space, while digital media is an uncertain multidimensional virtual space, which is based on the creation of four-dimensional space and time. Therefore, designers when conducting design thinking, we should convert the two-dimensional perspective to multidimensional and fully consider the expression of creativity in a three-dimensional way of thinking.

The relative inaccuracy reduces with increasing sample frequency. In comparison to SID and PBDCT, the relative error of the GPB technique is typically lower. Figures 6–8 display the relative inaccuracies of various test photos. It is evident that the GPB technique outperforms SID and PBD when recreating images at various sampling rates, demonstrating the algorithm's high levels of robustness and stability. The experimental findings demonstrate that the 3D image rebuilding system's overall impact is noticeably superior than the conventional 3D image rebuilding systems, and the antinoise ability has increased by 22.34%.

## 5. Reflections and Prospects of Visual Communication Design in the New Media Era

The contemporary visual transmission design has been significantly influenced by new media art. The resources employed in the design of visual transmission have increased with the gradual popularization of digital technology. Visual transmission design should get rid of the bondage of graphic design and meet the future of visual transmission design, but at the same time, visual transmission design also faces challenges. At present, the progress of emerging media technology needs to balance the relationship between science and technology and media. The interactive and high-tech characteristics of emerging media can stimulate the new ideas of visual transmission design, provide a platform for mutual communication for mass art, and promote the progress of visual transmission design.

1. Visual transmission design needs to pay more attention to the aesthetic feeling of design form. The visual transmission design under the emerging media technology has broken the time and space limitation once suffered in the traditional media and constructed a brand-new aesthetic paradigm in a brand-new context. In the emerging media, the dynamic visual expression of images and texts and the perceptual way of multisensory interaction are used to obtain a comprehensive experience, thus producing rich feelings and pleasure. With the continuous innovation and maturity of emerging media technology, visual transmission design needs to pay more attention to the aesthetic feeling of design form in order to meet the aesthetic needs of the public
2. In the emerging media environment, the innovation of traditional design concepts requires the continuous progress of emerging media art work, which has gradually developed from a single model in the past to a diversified model. In the actual design process, it is necessary to fully grasp people's daily life, so as to make the designed products more humanized, the works closer to reality, and meet people's psychological needs. The intuitiveness of visual transmission design should have obvious characteristics, but the traditional visual transmission design is not obvious in the form of expression, and it is relatively introverted, which hinders the progress of visual transmission design. The current visual transmission design is gradually integrated into humanistic care, so that the traditional visual transmission concept has been changed, and people can better accept the designed works, which is very beneficial to the progress of subsequent visual design
3. In terms of visual transmission on the emerging media interface, it is necessary to establish a mode of human-computer interaction. Visual transmission design has the characteristics of interactivity, which can meet the relevant needs of the audience for personalized information content to varying degrees. A high-quality interface makes it a pleasure to walk through, helping to facilitate the disappearance of the differences between the two worlds. It also changed the type of connection between the two worlds. Maybe the computer will never be able to realize the real interaction, but the novel visual design will make the communication between people and media more fit, complete, easy to operate, more dynamic, and interesting

## 6. Conclusion

The varied characteristics of visual transmission art practice activities at the form level and content level will gradually display a trend of varied progress and evolution with a relatively significant degree of expression against the backdrop of the increasingly sophisticated practice of emerging media technology. Additionally, it will, to a certain extent, bring about significant and profound changes in the fundamental assumptions underlying the practice of visual transmission art, which will have a significant and profound effect on the fundamental design tenets and fundamental design approaches of those activities. Design activity outcomes have drastically changed. All facets of visual transmission design have been greatly expanded with the development of the new media environment. Images, words, and sounds will all be included in the existing visual transmission system. To foster more dialogue and initiative in art design, designers use interactive and Internet technology. We should actively manage the current design staff and make an effort to do a good job at diversity control based on design application methods and selection of design expression elements if we want to achieve the best expected effect of visual transmission design against the backdrop of evolving media technology.

## Figures and Tables

**Figure 1:** Visual transmission technology system architecture.

**Figure 2:** Visual image processing process.

**Figure 3:** 3D rebuilding technology flow.

**Figure 4:** Variation of feature space parameters.

**Figure 5:** Weight parameter selection.

**Figure 6:** Image rebuilding quality impact under sampling data 1.

**Figure 7:** Image rebuilding quality impact under sampling data 2.

**Figure 8:** Image rebuilding quality effect under sampling data 3.

**Table 1:** Comparison results of different evaluation methods.

Reconstructed image	SNR	RLNE	*Ω*
Image 1	18.39	0.387	0.664
Image 2	19.28	0.987	0.388
Image 3	18.02	0.925	0.954

**Table 2:** Comparison of results under different division accuracy conditions.

Test subject	Division accuracy	3D image rebuilding time	Speedup ratio
Image A	0.238	18.37	1.49
	0.0294	63.29	10.47
	0.03458	32.389	13.45
Image B	3.288	18.9	1.587
	0.488	54.29	9.587
	0.579	43.398	12.598

## Data Availability

The data used to support the findings of this study are available from the corresponding author upon request.
